The article "Immediate versus Delayed Implantation for Single-Tooth Restoration of Maxillary Anterior Teeth: A Comparative Analysis on Efficacy" was published in 2022. Journal: Comput Math Methods Med.

# Immediate versus Delayed Implantation for Single-Tooth Restoration of Maxillary Anterior Teeth: A Comparative Analysis on Efficacy

**DOI:** 10.1155/2022/4490335

**Published:** 2022-06-09

**Authors:** Zhimin Chen, Shuhuai Zhang, Jun Zhou, Hongling Liang

**Affiliations:** Department of Stomatology, Suzhou Kowloon Hospital, Shanghai Jiaotong University School of Medicine, Suzhou, 215028 Jiangsu Province, China

## Abstract

**Objective:**

The present research is aimed at determining the efficacy of immediate implantation (II) and delayed implantation (DI) for single-tooth restoration of maxillary anterior teeth.

**Methods:**

From February 2019 to June 2020, 80 patients who received single-tooth restoration of maxillary anterior teeth in Suzhou Kowloon Hospital, Shanghai Jiaotong University School of Medicine, were included, among which 38 cases with DI restoration were used as the control group (CG), and the remaining 42 cases with II were used as the research group (RG). The complications that occurred were recorded. Besides, subjective satisfaction (Visual Analogue Scale (VAS)), aesthetic effect after anterior teeth trauma restoration (Pink Esthetic Score (PES)), aesthetics of dental hard tissue (White Esthetic Score (WES)), pocket depth assessed by pure titanium periodontal probe, implant stability (Implant Stability Quotient (ISQ)), and oral health-related quality of life (Oral Health Impact Profile- (OHIP-) 14) were evaluated. Attachment height, general look, color, and chewing function were all much higher in RG than in CG, according to the evaluation results. Furthermore, at 3 months, 6 months, and 12 months after surgery, RG had greater PES, WES, ISQ, and OHIP-14 scores, while the periodontal depth was decreased. In both groups of patients, the incidence of complications was similar, with no discernible differences.

## 1. Introduction

Tooth loss not only affects patients' facial aesthetics but also their chewing function, digestive function, and normal vocalization, resulting in a sharp decline in patients' quality of life (QOL). As the dental implant technology and biomaterials constantly develop, implant-supported dental restoration has become the first choice to replace missing teeth [1]. In the past, delayed implantation (DI) was mostly used; that is, implantation was accomplished 3 to 6 months after tooth extraction when the tooth extraction site was completely healed and the bone reconstruction was basically stable, so that the implant could form bony union after implantation with favorable safety [2]. However, this implant procedure will result in a protracted period of tooth loss, as well as keratinization of the gums and insufficient bone mass in the edentulous area due to alveolar bone absorption following tooth extraction, which will impact the aesthetic effect of implant repair [3, 4]. With the advances in stomatology, immediate implantation (II) technology has attracted the attention of stomatologists at home and abroad, as it not only shortens the number of surgical interventions and simplifies the treatment procedures but also preserves the soft tissue capsule to achieve the best soft tissue aesthetics [5, 6]. However, II is not omnipotent, and it will face challenges such as inadequate wound closure and insufficient soft tissue, which will greatly compromise the aesthetics of gingival formation of the implant in the aesthetic area [7]. In fact, the maxillary anterior teeth are very vulnerable to loss due to trauma or other causes given their special position. Once the maxillary anterior teeth are lost, it will not only affect patients' diet but also their appearance and image, seriously disturbing their normal life. At present, there are many comparative studies on II and DI restoration of single maxillary anterior teeth loss, but the comparison of soft tissue stability and aesthetics between the two implant restoration methods is relatively lacking. So we conducted this research for verification.

The article "Immediate versus Delayed Implantation for Single-Tooth Restoration of Maxillary Anterior Teeth: A Comparative Analysis on Efficacy" was published in 2022. Journal: Comput Math Methods Med.

The paper arrangements are as follows: Section 2 examines the data and methods.  Section 3 analyzes the result.  Section 4 discusses the discussion.  Section 5 concludes the work.

## 2. Data and Methods

This section discusses the research participants and evaluates the various treatment methods. They analyze the endpoint and discuss the statistical processing.

### 2.1. Research Participants

From February 2019 to June 2020, 80 patients who received single dental implant restoration of maxillary anterior teeth in Suzhou Kowloon Hospital, Shanghai Jiaotong University School of Medicine, were included as the research participants, among which 38 patients who used DI were taken as the control group (CG) and the remaining 42 patients who used II as the research group (RG). Inclusion criteria are as follows: age ≥ 18; single implant in the maxillary anterior region; good treatment compliance, oral hygiene, and oral care habits; sufficient bone mass at the implant site; no smoking history; healthy gums and stable occlusal relationship; no obvious periodontal inflammation; no contraindications for dental implants; and available bone height in the apical region of the teeth ≥ 3 mm, with no obvious soft and hard tissue defect. Exclusion criteria are as follows: inflammatory lesions in planting areas; prior bone augmentation surgery such as flap implantation; osteoporosis, diabetes, or other serious systemic diseases; and habitual grinding of teeth with severe symptoms. All subjects were informed and signed the informed consent. This study conforms to the Helsinki Declaration and is ethically ratified by Suzhou Kowloon Hospital, Shanghai Jiaotong University School of Medicine.

The article "Immediate versus Delayed Implantation for Single-Tooth Restoration of Maxillary Anterior Teeth: A Comparative Analysis on Efficacy" was published in 2022. Journal: Comput Math Methods Med.

### 2.2. Treatment

Periodontal tissue status, alveolar height, and alveolar bone width at the implant site were observed in both groups before surgery. Curved surface tomography and periapical film were taken and prepared before surgery, and the diameter and length of implants were determined. Antibiotics were prescribed half an hour prior to surgery.

#### 2.2.1. CG Was Treated with DI

Three months after extraction and exfoliation of the damaged anterior teeth, the absorption level of alveolar ridge and alveolar fossa healing was observed, and the implant restoration treatment was carried out only when the above two conditions were determined satisfactorily. Patients were placed in the supine position after receiving articaine for local anesthetic and following normal cleaning and towel laying. To thoroughly expose the implant area, a tiny incision was made from the crest of the alveolar ridge slightly to the palatal side, and the mucous bone flap was opened with a stripper. Then, with a torque of 35-50 N · cm, implants were routinely put, bone meal was implanted, and the surface was covered with a biofilm. Postoperatively, patients gargled with mouthwash and took antibiotics orally for 5-7 days. They were advised to return for a second-stage operation 5 months after the operation, and the full repair was carried out 2-3 months after the second-stage operation.

#### 2.2.2. RG Was Treated with II

Similarly, local anesthesia with articaine and routine disinfection and towel laying were performed before operation. The patient was placed in the supine position, and the small incision was made angular. The decision to extract the affected tooth or not was made depending on the periodontal wall condition and alveolar bone height. When designing the flap range of the incision, the integrity of the gingival papilla was tried to preserve as much as possible. The trauma caused by increased alveolar fossa was minimized during minimally invasive tooth extraction, and the integrity of bone wall was maintained. Then, the implant socket was prepared, and the suitable implant was determined, which was planted with a torque of ≥35 N · cm, reaching at least 3.0-5.0 mm at the bottom of alveolar socket as the implant depth and reserving a tongue-labial bone wall with a thickness of more than 1.0 mm. The implant's crown square was about 0.5 mm smaller than the bottom of the alveolar socket, which was consistent with the long axis of the opposite side. The surface was then covered with biofilm, and bone meal was implanted in the space around the implant. According to the position of the missing teeth and the size of adjacent teeth, the specifications and models of the immediate implant abutment were determined, and nanoresin was used as temporary crown. After abutment implantation, attention was paid to tight suture, and the neck of abutment was highly polished to ensure no occlusal contact. Besides, the anterior, lateral, and median of the abutment were adjusted, after which central screws were used for fixation. After the operation, patients were gargled with mouthwash, and oral antibiotics were taken for 7 days. The full crown restoration was completed 6 months after surgery.

The article "Immediate versus Delayed Implantation for Single-Tooth Restoration of Maxillary Anterior Teeth: A Comparative Analysis on Efficacy" was published in 2022. Journal: Comput Math Methods Med.

### 2.3. Endpoints

#### 2.3.1. Success Rate of Restoration

Adequate periodontal tissue, no loosening of implants, and normal chewing function were all criteria for restoration success. Repair failure was defined as gingival periodontal redness and abscess, implant loosening, and no improvement or even deterioration of chewing ability following therapy. Besides, the common complications of dental implantation in both groups were recorded, including gingival margin recession, peri-implant inflammation, metal exposure, and infection.

Subjective satisfaction was assessed 1 year after surgery based on patients' subjective feelings using the Visual Analogue Scale (VAS). The indexes include attachment height, overall appearance, color, and chewing function. Satisfaction is positively correlated with the score (range: 0-10).

The Pink Esthetic Score (PES) [8] was used to evaluate the aesthetic effect of patients after the anterior tooth restoration, which was evaluated once at 3 months, 6 months, and 12 months after the operation, with a total of 7 items and 0-2 points for each item. The aesthetics of tooth hard tissue was assessed using the White Esthetic Score (WES) [9] from five domains of color, surface texture, tooth form, tooth volume/outline, and translucency, and each item scored 0-2 points. For both scales, higher scores are associated with better aesthetic effects.

A pure titanium periodontal probe was used to detect the pocket depth (PD) at 3 months, 6 months, and 12 months postoperatively, and the detection position was the distance between the pocket bottom of the implant denture and the mesial, central, and distal gingival margins on the labial and lingual surfaces of the crowns. Implant stability was assessed using the Implant Stability Quotient (ISQ) [10] (score range: 0-100), with higher scores indicating better implant stability.

The article "Immediate versus Delayed Implantation for Single-Tooth Restoration of Maxillary Anterior Teeth: A Comparative Analysis on Efficacy" was published in 2022. Journal: Comput Math Methods Med.

The evaluation of oral health-related QOL at 3, 6, and 12 months after surgery employed the Oral Health Impact Profile- (OHIP-) 14 scales [11]. The scale includes 7 dimensions with 2 items each, and the score of each item is 0-4 points, with a total score of 0-56 points. The higher the score, the lower the QOL related to oral health.

### 2.4. Statistical Processing

Data were statistically processed by SPSS 19.0 (Shanghai Yijun Information Technology) and visualized into figures via GraphPad Prism 6. Chi-square test and independent *t*-test were applied for comparison of counting data and measurement data in this paper, respectively, with the threshold of significance set as *P* < 0.05.

## 3. Results

Here, it examines the comparison of general data and occurrence of complications. We analyzed the comparison of attachment height, overall appearance, color, and masticatory function and define the PES and WES scores of patients in two groups at different time points. We also discussed the PD and ISQ scores at different time points in two groups and oral health-related QOL.

### 3.1. Comparison of General Data

General data like sex, age, BMI, educational level, and causes of tooth loss showed no distinct differences between RG and CG (*P* > 0.05) (Table 1).

### 3.2. Occurrence of Complications

The common complications of dental implant in the two groups were recorded. In CG, gingival margin recession, peri-implant inflammation, metal exposure, and infection were observed in 2 (5.26%), 1 (2.63%), 2 (5.26%), and 0, respectively, with an overall incidence of 13.16%. While in RG, the data were 2 (4.76%), 1 (2.38%), 1 (2.38%), and 1 (2.38%), respectively, and the total incidence was 11.90%. Complications were similar between the two groups with no significant difference (*P* > 0.05) nor was there any notable difference in the success rate of repair between RG and CG after statistical analysis (97.62% vs. 94.74%, *P* > 0.05) (Table 2).

### 3.3. Comparison of Attachment Height, Overall Appearance, Color, and Masticatory Function

The results of patients' subjective satisfaction evaluated by VAS showed that the attachment height, overall appearance, color, and chewing function were significantly higher in RG than in CG (*P* < 0.05) (Table 3).

### 3.4. PES and WES Scores of Patients in Two Groups at Different Time Points

PES and WES were used to evaluate the improvement of the aesthetic effect. The data revealed higher PES and WES scores in RG compared with CG at 3 months, 6 months, and 12 months after surgery (*P* < 0.05) (Figure 1).

### 3.5. PD and ISQ Scores at Different Time Points in Two Groups

Compared with CG, the PD in RG decreased significantly at 3 months, 6 months, and 12 months after surgery, while the ISQ score increased significantly (*P* < 0.05) as shown in Figure 2.

The article "Immediate versus Delayed Implantation for Single-Tooth Restoration of Maxillary Anterior Teeth: A Comparative Analysis on Efficacy" was published in 2022. Journal: Comput Math Methods Med.

### 3.6. Oral Health-Related QOL

The oral health-related QOL assessed by OHIP-14 scale determined higher scores in RG compared with CG at 3 months, 6 months, and 12 months after surgery (*P* < 0.05) (Figure 3).

## 4. Discussion

The results of this study support the use of II as the preferred method of dental restoration for patients with single maxillary anterior teeth loss, as it provides better aesthetic support with higher treatment satisfaction, implant stability, and QOL compared to DI.

The teeth between the canines on both sides of the maxilla are known as maxillary anterior teeth. Losing anterior teeth will compromise the patient's physiological functions like as chewing and speech, as well as their overall looks, causing major negative effects on their physical and mental health and daily lives. At present, single-tooth implants have a good long-term survival rate, but implantation remains challenging due to the frequent presence of hard and soft tissue resorption defects and the high aesthetic requirements of the aesthetic area [12]. DI is a mature and reliable means of conventional plant restoration. Patients must, however, wait for the wound to heal following tooth extraction, and the resulting long period of time without teeth will damage their appearance and daily lives, putting a psychological and financial strain on the patients. Therefore, patients with anterior tooth loss will have certain concerns when choosing DI. II, on the other hand, can avoid the above shortcomings of DI [13, 14], but its influence on the aesthetic appearance of patients is controversial. Some studies suggest that II is not aesthetically friendly to patients [15, 16]. While some other evidence argues that II has similar effects and is even superior to DI on patients' aesthetic appearance [17–19]. In this study, RG showed better performance in the evaluation of attachment height, overall appearance, color, and chewing function, with higher PES and WES scores than CG at 3 months, 6 months, and 12 months after surgery, which shows that II is more esthetically pleasing. The reason may be that II can reduce and avoid alveolar bone absorption, better maintain soft tissue morphology, and effectively maintain the height and width as well as the physiological stimulation of the alveolar bone, thus achieving the aesthetic effect that DI cannot achieve [20].

It is shown that the success rate of II and DI is comparable, usually above 90% [21, 22]. The results of this study also found that the success rate of the two plantation methods exceeded 90% with no significant difference. Following that, we discovered no statistically significant difference in the occurrence of problems between the two groups. However, when compared to CG, RG's PD fell dramatically at 3 months, 6 months, and 12 months following surgery, while the ISQ score climbed significantly. These findings show that both implantation procedures are feasible and safe for single-tooth maxillary anterior tooth repair. However, II better facilitates the formation of good periodontal attachment, provides favorable support conditions for the growth of attached gingiva, and protects the alveolar bone septum, playing a more significant role than DI in promoting the health of patients' periodontal tissue.

The article "Immediate versus Delayed Implantation for Single-Tooth Restoration of Maxillary Anterior Teeth: A Comparative Analysis on Efficacy" was published in 2022. Journal: Comput Math Methods Med.

Due to the destruction of dental integrity, patients with tooth loss may suffer from alveolar bone atrophy, decreased masticatory function, food impaction, adjacent tooth displacement, and mandibular joint lesions, which may have adverse effects on patients' physiological function and psychological state, seriously affecting their QOL [23, 24]. Therefore, oral health-related QOL is one of the most important indicators to evaluate the success of implantation and restoration. In this study, the OHIP-14 scale was used to evaluate the influence of II and DI on patients' oral-related QOL. At 3, 6, and 12 months following surgery, RG had considerably higher OHIP-14 scores than CG, indicating that II could significantly enhance patients' oral-related QOL. This could be due to the fact that II minimizes the duration of missing teeth and the number of follow-up visits, eliminates aesthetic and pronunciation issues, and eliminates psychological and social barriers, all of which improve patients' QOL greatly.

## 5. Conclusions

Without causing major complications, II contributes to better aesthetic effects, higher subjective satisfaction, and superior postoperative quality of life for patients with single-tooth restoration of maxillary anterior teeth, which is worth for clinical use. For patients with single maxillary anterior tooth loss, II has higher prognostic value and is more conducive to improving implant stability, treatment satisfaction, and QOL with more significant aesthetic effects, which is worth promoting clinically.

## Figures and Tables

**Figure 1:** PES and WES scores of patients in two groups at different time points. (a) The PES scores of the research group at 3 months, 6 months, and 12 months after surgery were higher than those of the control group. (b) The WES scores of the research group at 3 months, 6 months, and 12 months after surgery were higher than those of the control group. ^∗^ represents *P* < 0.05 compared with the control group at the same time point.

The article "Immediate versus Delayed Implantation for Single-Tooth Restoration of Maxillary Anterior Teeth: A Comparative Analysis on Efficacy" was published in 2022. Journal: Comput Math Methods Med.

**Figure 2:** Pocket depth and ISQ score of two groups of patients at different time points. (a) The pocket depth of the research group was lower than that in the control group at 3 months, 6 months, and 12 months after surgery. (b) The ISQ score of the research group was higher than that of the control group at 3, 6, and 12 months after surgery. ^∗^ represents *P* < 0.05 compared with the control group at the same time point.

**Figure 3:** Oral health-related quality of life. The total score of OHIP-14 in the research group at 3 months, 6 months, and 12 months after surgery was significantly higher than that in the control group. ^∗^ represents *P* < 0.05 compared with the control group at the same time point.

**Table 1:** Comparison of general data between two groups of patients.

Groups	Control group (*n* = 38)	Research group (*n* = 42)	*χ* ^2^/*t*	*P*
Sex			0.637	0.425
Male	23 (60.53)	29 (69.05)		
Female	15 (39.47)	13 (30.95)		
Age (years old)	33.21 ± 9.56	33.98 ± 9.83	0.724	0.355
BMI (kg/m^2^)	22.93 ± 1.33	23.12 ± 1.56	0.583	0.562
Educational level			1.229	0.268
≥High school	17 (44.74)	24 (57.14)		
<High school	21 (55.26)	18 (42.86)		
Causes of tooth loss			2.036	0.361
Caries	13 (34.21)	11 (26.19)		
Trauma	13 (34.21)	21 (50.00)		
Others	12 (31.58)	10 (23.81)		

**Table 2:** Occurrence of complications.

Groups	Control group (*n* = 38)	Research group (*n* = 42)	*χ* ^2^	*P*
Gingival margin recession	2 (5.26)	2 (4.76)		
Peri-implant inflammation	1 (2.63)	1 (2.38)		
Metal exposure	2 (5.26)	1 (2.38)		
Infection	0 (0.00)	1 (2.38)		
Total	5 (13.16)	5 (11.90)	0.03	0.87
Success rate of repair	36 (94.74)	41 (97.62)	0.46	0.49

**Table 3:** Comparison of attachment height, overall appearance, color, and masticatory function between the two groups.

Groups	Control group (*n* = 38)	Research group (*n* = 42)	*t*	*P*
Attachment height	7.26 ± 1.06	8.02 ± 1.42	2.690	0.009
Overall appearance	7.05 ± 1.11	7.79 ± 1.30	2.724	0.008
Color	7.42 ± 1.06	8.12 ± 1.38	2.524	0.014
Masticatory function	6.97 ± 1.08	7.55 ± 1.33	2.127	0.037

## Data Availability

The labeled datasets used to support the findings of this study are available from the corresponding author upon request.

## References

[1] Wu D., Zhou L., Lin J., Chen J., Huang W., Chen Y. (2019). Immediate implant placement in anterior teeth with grafting material of autogenous tooth bone vs xenogenic bone. *BMC Oral Health*.

[2] Meng W., Chien Y., Chien H. (2021). Immediate implant placement and provisionalization in the esthetic zone: a 6.5-year follow-up and literature review. *Case Reports in Dentistry*.

[3] Cosyn J., De L., Seyssens L., Doornewaard R., Deschepper E., Vervaeke S. (2019). The effectiveness of immediate implant placement for single tooth replacement compared to delayed implant placement: a systematic review and meta-analysis. *Journal of Clinical Periodontology*.

The article "Immediate versus Delayed Implantation for Single-Tooth Restoration of Maxillary Anterior Teeth: A Comparative Analysis on Efficacy" was published in 2022. Journal: Comput Math Methods Med.

[4] Aldhohrah T., Qin G., Liang D. (2022). Does simultaneous soft tissue augmentation around immediate or delayed dental implant placement using sub-epithelial connective tissue graft provide better outcomes compared to other treatment options? A systematic review and meta-analysis. *PLoS One*.

[5] Saijeva A., Juodzbalys G. (2020). Immediate implant placement in non-infected sockets versus infected sockets: a systematic review and meta-analysis. *Journal of oral & maxillofacial research*.

[6] Amin V., Kumar S., Joshi S., Hirani T., Shishoo D. (2019). A clinical and radiographical comparison of buccolingual crestal bone changes after immediate and delayed implant placement. *Medicine and Pharmacy Reports*.

[7] Fang J., Xin R., Li W., Wang C., Lv X., Zhou M. (2021). Immediate implant placement in combination with platelet rich-fibrin into extraction sites with periapical infection in the esthetic zone: a case report and review of literature. *World Journal of Clinical Cases*.

[8] Furhauser R., Florescu D., Benesch T., Haas R., Mailath G., Watzek G. (2005). Evaluation of soft tissue around single-tooth implant crowns: the pink esthetic score. *Clinical Oral Implants Research*.

[9] Chen J., Chiang C., Zhang Y. (2018). Esthetic evaluation of natural teeth in anterior maxilla using the pink and white esthetic scores. *Clinical Implant Dentistry and Related Research*.

[10] Levin P. (2016). The correlation between immediate implant insertion torque and implant stability quotient. *The International Journal of Periodontics & Restorative Dentistry*.

[11] Slade D. (1997). Derivation and validation of a short-form oral health impact profile. *Community Dentistry and Oral Epidemiology*.

[12] Afrashtehfar I., Assery A., Bryant R. (2021). Aesthetic parameters and patient-perspective assessment tools for maxillary anterior single implants. *International journal of dentistry*.

[13] Bassir H., Kholy K., Chen Y., Lee H., Intini G. (2019). Outcome of early dental implant placement versus other dental implant placement protocols: a systematic review and meta-analysis. *Journal of Periodontology*.

[14] Arora H., Ivanovski S. (2018). Clinical and aesthetic outcomes of immediately placed single-tooth implants with immediate vs. delayed restoration in the anterior maxilla: a retrospective cohort study. *Clinical Oral Implants Research*.

[15] Cosyn J., Eghbali A., Hermans A., Vervaeke S., Bruyn H., Cleymaet R. (2016). A 5-year prospective study on single immediate implants in the aesthetic zone. *Journal of Clinical Periodontology*.

The article "Immediate versus Delayed Implantation for Single-Tooth Restoration of Maxillary Anterior Teeth: A Comparative Analysis on Efficacy" was published in 2022. Journal: Comput Math Methods Med.

[16] Tonetti S., Cortellini P., Graziani F. (2017). Immediate versus delayed implant placement after anterior single tooth extraction: the timing randomized controlled clinical trial. *Journal of Clinical Periodontology*.

[17] Buser D., Chappuis V., Bornstein M., Wittneben G., Frei M., Belser C. (2013). Long-term stability of contour augmentation with early implant placement following single tooth extraction in the esthetic zone: a prospective, cross-sectional study in 41 patients with a 5- to 9-year follow-up. *Journal of Periodontology*.

[18] Arora H., Ivanovski S. (2018). Evaluation of the influence of implant placement timing on the esthetic outcomes of single tooth implant treatment in the anterior maxilla: a retrospective study. *Journal of Esthetic and Restorative Dentistry*.

[19] Canellas J., Medeiros D., Figueredo C., Fischer G., Ritto G. (2019). Which is the best choice after tooth extraction, immediate implant placement or delayed placement with alveolar ridge preservation? A systematic review and meta-analysis. *Journal of Cranio-Maxillo-Facial Surgery*.

[20] Mahesh L., Calvo L., Shukla S., Kumar R., Kumar R. (2020). Clinical and radiographic findings without the use of bone substitute materials in extraction sockets and delayed implant placement- a case series. *Journal of Oral Biology and Craniofacial Research*.

[21] Thanissorn C., Guo J., Jing D. (2022). Success rates and complications associated with single immediate implants: a systematic review. *Dentistry Journal*.

[22] Smith B., Tarnow P., Sarnachiaro G. (2019). Immediate placement of dental implants in molar extraction sockets: an 11-year retrospective analysis. *The Compendium of Continuing Education in Dentistry*.

[23] Khan U., Ghani F., Nazir Z. (2018). The effect of some missing teeth on a subjects’ oral health related quality of life. *Pakistan Journal of Medical Sciences*.

[24] Schierz O., Baba K., Fueki K. (2021). Functional oral health-related quality of life impact: a systematic review in populations with tooth loss. *Journal of Oral Rehabilitation*.

